# Diagnosis of transition zone prostate cancer by multiparametric MRI: added value of MR spectroscopic imaging with sLASER volume selection

**DOI:** 10.1186/s12929-021-00750-6

**Published:** 2021-07-19

**Authors:** Neda Gholizadeh, Peter B. Greer, John Simpson, Jonathan Goodwin, Caixia Fu, Peter Lau, Saabir Siddique, Arend Heerschap, Saadallah Ramadan

**Affiliations:** 1 School of Health Sciences, Faculty of Health and Medicine, University of Newcastle, Newcastle, NSW Australia; 2 School of Mathematical and Physical Sciences, University of Newcastle, Newcastle, NSW Australia; 3 Calvary Mater Newcastle, Radiation Oncology Department, Newcastle, NSW Australia; 4 MR Application Development, Siemens Shenzhen Magnetic Resonance Ltd., Shenzhen, China; 5 Radiology Department, Calvary Mater Newcastle, Newcastle, NSW Australia; 6 Hunter Medical Research Institute (HMRI) Imaging Centre, New Lambton Heights, NSW Australia; 7 Department of Radiology and Nuclear Medicine, Radboud University Medical Center, Nijmegen, The Netherlands

**Keywords:** Prostate cancer, Multiparametric MRI, ^1^H MR spectroscopic imaging, GOIA-sLASER, SVM

## Abstract

**Background:**

Current multiparametric MRI (mp-MRI) in routine clinical practice has poor-to-moderate diagnostic performance for transition zone prostate cancer. The aim of this study was to evaluate the potential diagnostic performance of novel ^1^H magnetic resonance spectroscopic imaging (MRSI) using a semi-localized adiabatic selective refocusing (sLASER) sequence with gradient offset independent adiabaticity (GOIA) pulses in addition to the routine mp-MRI, including T2-weighted imaging (T2WI), diffusion-weighted imaging (DWI) and quantitative dynamic contrast enhancement (DCE) for transition zone prostate cancer detection, localization and grading.

**Methods:**

Forty-one transition zone prostate cancer patients underwent mp-MRI with an external phased-array coil. Normal and cancer regions were delineated by two radiologists and divided into low-risk, intermediate-risk, and high-risk categories based on TRUS guided biopsy results. Support vector machine models were built using different clinically applicable combinations of T2WI, DWI, DCE, and MRSI. The diagnostic performance of each model in cancer detection was evaluated using the area under curve (AUC) of the receiver operating characteristic diagram. Then accuracy, sensitivity and specificity of each model were calculated. Furthermore, the correlation of mp-MRI parameters with low-risk, intermediate-risk and high-risk cancers were calculated using the Spearman correlation coefficient.

**Results:**

The addition of MRSI to T2WI + DWI and T2WI + DWI + DCE improved the accuracy, sensitivity and specificity for cancer detection. The best performance was achieved with T2WI + DWI + MRSI where the addition of MRSI improved the AUC, accuracy, sensitivity and specificity from 0.86 to 0.99, 0.83 to 0.96, 0.80 to 0.95, and 0.85 to 0.97 respectively. The (choline + spermine + creatine)/citrate ratio of MRSI showed the highest correlation with cancer risk groups (r = 0.64, p < 0.01).

**Conclusion:**

The inclusion of GOIA-sLASER MRSI into conventional mp-MRI significantly improves the diagnostic accuracy of the detection and aggressiveness assessment of transition zone prostate cancer.

## Background

Prostate cancer (PCa) is the most common malignancy and the fourth leading cause of cancer death among males worldwide [1]. Almost 30% of PCa lesions occur in the transition zone (TZ) [2]. TZ cancer has a relatively low Gleason score (GS), local stage and biochemical recurrence rate in comparison with peripheral zone (PZ) PCa [3]. Due to difficulties in localizing TZ by digital rectal exam, sampling of TZ cancer by routine transrectal ultrasound (TRUS)-guided biopsy and low specificity of prostate specific antigen (PSA) as cancer marker, there is a high potential risk for missing TZ lesions [4]. Magnetic resonance imaging (MRI) with its non-invasive soft tissue contrast capability has the potential to overcome these limitations for the detection of TZ cancer [5]. T2-weighted imaging (T2WI) provides the best anatomical images of TZ and PZ. However, TZ often contains benign prostatic hyperplasia (BPH), which may have low-signal intensity on T2WI similar to that of cancer [6]. Furthermore, the clinical application of multiparametric MRI (mp-MRI) including T2WI, diffusion-weighted imaging (DWI) and dynamic contrast enhanced (DCE) imaging as defined by the Prostate Imaging Reporting and Data System (PI-RADS V2) has shown moderate diagnostic performance for TZ cancer [7]. The overlap of apparent diffusion coefficient (ADC) values between cancer and BPH in TZ is the main limitation of DWI [8]. DCE has a minor role in TZ cancer detection because BPH in TZ can be highly vascularized and shows rapid and high level enhancement similar to PCa [9]. The diagnostic potential of proton MR spectroscopic imaging (MRSI) in combination with anatomical and functional MRI for the improvement of PCa detection, localization and characterization has already been demonstrated [10, 11]. Point-resolved spectroscopy (PRESS) is the most commonly used pulse sequence for prostate MRSI mainly because of its commercial availability, but it suffers from chemical shift displacement error, long acquisition time and bad slice profiles, which causes unpredictable lipid signal contamination. These problems were addressed by using a semi-localized adiabatic selective refocusing pulse sequence (sLASER) with gradient-modulated offset-independent adiabatic (GOIA) pulses (GOIA-sLASER), which resulted in much cleaner MR spectra of the prostate [12]. To our knowledge, there have been no reports on the diagnostic performance of MRSI GOIA-sLASER within routine clinical prostate mp-MRI exams.

The purpose of this study was to evaluate the diagnostic performance of individual and combined mp-MRI parameters, employed for PI-RADS evaluations, and GOIA-sLASER MRSI using an external phased-array coil for TZ cancer detection, localization and grading.

## Methods

### Patients

In total, 45 patients with biopsy-proven TZ cancer and one biopsy-negative subject were consecutively enrolled in this study. Four patients were excluded from the study due to poor-quality data. The study protocol was approved by the local Human Research Ethics Committee and each patient signed a consent form before the MRI examination. Depending on prostate gland size, at least sixteen TRUS guided biopsy cores were obtained from each patient between six to eight weeks before the MRI examination.

### MRI acquisition protocol

Prostate mp-MRI was performed on a whole-body 3 T MR scanner using an eighteen-channel phased-array coil (MAGNETOM Prisma, Siemens Healthcare, Erlangen, Germany) and without endorectal coil. The mp-MRI protocol included axial, coronal and sagittal T2WI, DWI and three-dimensional (3D) MRSI. The last step in this protocol was DCE MRI for which paramagnetic gadolinium (Gadovist®, Bayer Heathcare Pharmaceuticals, Berlin, Germany) was administered as bolus injection of 0.1 mmol/kg body weight with a power injector at 2.5 mL/s and followed by a 15-mL saline flush. A DCE time series was acquired with a T1-weighted sequence including 4 baseline acquisitions before the injection. Details of the mp-MRI acquisition parameters are summarized in Table 1.

**Table 1:** MRI acquisition parameters for prostate multiparametric MRI (mp-MRI)

	T2WI (Axial)	T2WI (Coronal)	T2WI (Sagittal)	DWI	DCE	MRSI
Sequence	2D TSE	2D TSE	2D TSE	EPI	3D VIBE	GOIA-sLASER
TR (ms)	4300	3620	4500	3400	4.88	820
TE (ms)	102	104	90	53	1.77	88
Averages	2	3	3	16	1	4
Flip angle (degree)	160	160	128	90	15	90–4 × 180
Thickness (mm)	3	3	3	3	3	7
Gap (mm)	0	0	0	0	0	0
FOV (mm)	200 × 200	200 × 200	240 × 240	256 × 256	260 × 260	84 × 84 × 70
b-value (s/mm^2^)	NA	NA	NA	0, 400, 800 and 1600	NA	NA
Temporal resolution (s)	NA	NA	NA	NA	4.8	NA
Matrix	448 × 448 × 30	448 × 448 × 30	320 × 320 × 24	84 × 128 × 24	192 × 192 × 24	12 × 12 × 10
Spatial resolution (mm^3^)	0.45 × 0.45 × 3	0.45 × 0.45 × 3	0.75 × 0.75 × 3	2 × 2 × 3	1.35 × 1.35 × 3	7 × 7 × 7
Acquisition time (min)	3.19	4.51	4.05	6.26	6.23	8.42

*TR* repetition time, *TE* echo time, *FOV* field of view, *TSE* turbo spin echo, *EPI* echo planar imaging, *VIBE* volumetric interpolated breath-hold examination, *GOIA-sLASER* gradient offset independent adiabaticity with semi-localized adiabatic selective refocusing, *NA* not available/not applicable

### MRI prostate mapping and pre-processing

Bias correction, noise reduction and intensity standardisation were applied on T2WI [13].

ADC maps were calculated inline from DWI’s using a mono-exponential fitting of b-values 0, 400, 800 and 1600 s/mm^2^ in syngo software.

DCE-MR images were processed by a Siemens dedicated Tissue4D module for dynamic analysis of DCE MR with an implementation of the Tofts model and an assumed arterial input function (AIF) [14]. After motion correction, optimal AIFs were selected from slow, intermediate and fast population-averaged options, considering individual volume of interest (VOI) curves. The quantitative variables derived from T1 maps were the volume transfer constant (K^trans^, min^−1^), the rate constant (K_ep_, min^−1^) and the area under gadolinium curve (iAUGC, mmol min/L).

Citrate (Cit), creatine (Cr), choline (Cho) and spermine (Spm) tissue concentrations within a voxel were determined by the automated peak fitting algorithm LCModel (Version 6.3-1L) using metabolite basis sets. Two Cit ratios, ((Cho + Spm + Cr)/Cit and Cho/Cit), and the Cho/Cr ratio were calculated for each voxel within a selected region (vide infra).

### Tissue segmentation

All patients underwent at least 16-core (S16C) transrectal and transperineal ultrasound-guided biopsy using a reusable biopsy gun. Two independent radiologists, one with more than twenty years’ experience (P.L.) and one with thirteen years’ experience (S.S.) in prostate radiology, evaluated all MRI images in conjunction with the biopsy reported cancer locations. Radiologists visually matched ADC maps, baseline images (b-value = 0 s/mm^2^), and corresponding T2WI slice locations and gland anatomy (apex, mid-gland area and base).

In total, 61 cancer regions with biopsy-proven positive TZ cancer (1–3 cancer regions per patient) were manually delineated on T2WI by the two radiologists and these were subsequently co-registered to the corresponding ADC, DCE and MRSI maps. To maximize the identification accuracy of the cancer regions, only concurrent reporting of cancer ROIs was used. Then, the two radiologists in consensus selected 73 normal regions from TZ with negative biopsies (1–2 normal regions per patient). Each cancer or normal region was selected over one ROI on a single slice or multiple ROIs on multiple slices for each patient. The ROIs on multiple slices for each tissue were summarised per mean value to eliminate bias.

### Assessment of histologic tumor grade

Cancerous tissues were sub-divided according to GS into three main risk groups to evaluate the value of mp-MRI parameters to discriminate between different cancer grades. These risk groups are (a) 37 regions with GS of 3 + 3 as low-risk, (b) 9 regions with GS of 3 + 4 as intermediate-risk and (c) 15 regions with GS ≥ 4 + 3 as high-risk. Each cancer region parameter on mp-MRI maps was subsequently correlated to the matching GS group based on biopsy results.

### Classification and statistical analysis

A non-parametric Mann–Whitney U-test with Bonferroni correction was performed for each pair group to determine significant difference between the mean values of normal and cancer regions of mp-MRI parameters.

We developed a machine learning platform for mp-MRI including support vector machine (SVM) classifications with a radial basis function kernel (RBF-SVM) and area under receiver operator characteristic (ROC) analyses using an in-house Matlab routine to evaluate the diagnostic performance of models with different parametric combinations: T2WI + DWI, T2WI + DWI + DCE, T2WI + DWI + MRSI, and T2WI + DWI + DCE + MRSI. Mp-MRI parameters involved were ADC, K^trans^, K_ep_, iAUGC, (Cho + Spm + Cr)/Cit, Cho/Cit and Cho/Cr. Models were developed with mp-MRI parameters with a statistically significant difference between each pair group. The sensitivity, specificity and overall accuracy of each classifier are reported.

The correlation between risk groups (low-risk, intermediate-risk and high-risk) and mp-MRI parameters was measured with Spearman correlation coefficient (r) (IBM SPSS). Then, mp-MRI parameters with |r|≥ 0.25 were used to develop RBF-SVM models between cancer risk groups. These models were used to evaluate the diagnostic performance of mp-MRI parameters to differentiate cancer risk groups. All evaluations were based on biopsy results.

Optimal kernel parameters for RBF-SVM were calculated by a grid search approach [15]. The performance of the SVM classification models was determined by leave-one-out cross-validation.

McNemar tests were used for pairwise comparisons of sensitivity and specificity between different mp-MRI models, while Delong test was used to compare the area under curves (AUCs). A *p* value < 0.05 was considered statistically significant.

## Results

### Multiparametric MRI of prostate cancer patients

To avoid inclusion of low-quality data, the MR data from four patients were excluded from the study as they showed distortion artefacts on DWI and had a FWHM_water_ > 50 Hz for the whole prostate gland, related to patients’ movements and motion during scanning. Clinical and demographic data of the remaining 41 patients are summarized in Table 2.

**Table 2:** Demographic and clinical data of the prostate cancer patients enrolled in this study (A) and Gleason score of biopsies (B)

A)	Mean ± SD	Range
Age (years)	66.31 ± 7.19	53 – 81
PSA (ng/mL)	7.82 ± 3.91	2.5 – 18.9
Prostate volume (cm^3^)	45.01 ± 17.23	22.02 – 91.11

B) Biopsy Gleason Score	Number of biopy-proven cancer tissue (total = 61)	% of total
3 + 3	37	60.7
3 + 4	9	14.7
4 + 3	7	11.5
4 + 4	6	9.8
4 + 5	2	3.3

*PSA* prostate specific antigen

Employing a phased-array receive coil (without an endorectal coil), the application of GOIA-sLASER MRSI to the prostate produced MR spectra showing well-resolved metabolite signals with adequate SNR (Figs. 1G, 2G and 3G).

**Fig. 1:** Multiparametric MRI of the prostate of a 58-year-old man with an elevated serum PSA level of 6.8 ng/mL and cancer-negative biopsy results. **A** T2WI with low-signal intensity areas in the left and right transition zone (arrows) which were biopsy negative for cancer. **B** ADC map showing low-signal intensity for the same areas. High-signal intensity for these areas were seen on **C** high b-value DWI and on pharmacokinetic maps of **D** K^trans^, **E** K_ep_, and **F** iAUGC. **G** Middle: MRSI grid and color-coded map overlaid on T2WI. The spectra in the yellow box at the right side and in the green box at the left side represent voxels from histopathology confirmed normal tissue (circles)

**Fig. 2:** Multiparametric MRI of the prostate of a 68-year-old man with a serum PSA level of 4.3 ng/ml, who was diagnosed with a biopsy-proven Gleason 3 + 3 cancer region in the left of the transition zone (arrows). The area on the right of the transition zone (arrows) had a cancer-negative biopsy outcome. **A** T2WI, **B** ADC map, **C** high b-value DWI, pharmacokinetic maps of calculated **D** K^trans^, **E** K_ep_, **F** iAUGC and **G** MRSI grid and color-coded map overlaid on T2WI, with the red circle representing a voxel with cancer (spectrum in box at the left hand side) and the green circle representing a voxel with normal tissue (spectrum in box at the right hand side)

**Fig. 3:** Multiparametric MRI of the prostate of a 59-year-old patient with an elevated serum PSA level of 12.1 ng/ml, who was diagnosed with a biopsy-proven prostate cancer with Gleason 4+4 in the right side of the transition zone (arrows). **A** T2WI, **B** ADC map, **C** high b-value DWI, and pharmacokinetic maps of **D** K^trans^, **E** K_ep_,and **F** iAUGC. **G** MRSI grid and color-coded map of (Cho + Spm + Cr)/Cit values overlaid on T2WI, with red circle identifying a voxel in cancer region and green circle for a voxel in normal tissue. Left: MR spectrum from voxel of cancer tissue spectrum (red box). Right: MR spectrum from voxel of normal tissue (green box)

Figure 1 shows MR data of a prostate which was biopsy-proven negative for PCa. The negative-biopsy areas in the left and right TZ appeared as low-signal intensity on T2WI and the ADC map (restricted diffusion) and as high-signal intensity on high b-value DWI, K^trans^ and iAUGC maps (Fig. 1A–D, F). However, these areas appeared as normal on K_ep_ maps (Fig. 1E). Moreover, the MR spectra, derived from the MRSI exam, of these (biopsy cancer negative) ROIs exhibited high Cit and low Cho signals (Fig. 1G) representing normal prostate tissue and thus providing vital information indicative of the absence of cancer tissue.

Figure 2 shows data of an mp-MRI exam obtained from a patient with a region in the prostate with low-risk cancer (GS = 3 + 3) in the left TZ ( arrows). This region appeared as low-signal intensity on T2WI and on the ADC map (Fig. 2A, B) and high-signal intensity on high b-value DWI and on pharmacokinetic maps derived from DCE (Fig. 2C–F). The MR spectra obtained from this ROI exhibited relatively high Cho signals and low Cit signals (Fig. 2G, right). A negative biopsy area in the right TZ of the prostate of this patient (arrows) also appeared as low-signal intensity on T2WI and the ADC map (restricted diffusion) and as high-signal intensity on high b-value DWI and pharmacokinetic maps (Fig. 2A–F), all suggesting the presence of cancer tissue. However, the MR spectra of this region, derived from the 3D MRSI exam, exhibited normal high Cit signals and low Cho signals (Fig. 2G, left), in complete agreement with the biopsy results that this region contains no cancer.

In patients with high-risk TZ prostate cancers, tumor tissue presented as low-signal intensity on T2WI and ADC maps and high-signal intensity on high b-value DWI and pharmacokinetic parameter maps of DCE exams (Fig. 3A–F). Normal TZ tissue showed higher signal intensity on ADC maps (Fig. 3B). However, quantitative DCE parameters maps generally showed inconclusive enhancements making them ineffective in the differentiation of central cancer tissue from normal tissue. MRSI spectral maps of the entire prostate showed low-signal intensity levels for Cit and high-intensity levels for Cho in tumor areas (Fig. 3G, left), whereas normal TZ tissue showed relatively high levels of Cit and low levels of Cho (Fig. 3G, right).

In addition, in five patients with both TZ and PZ PCa, high quality MR spectra were obtained for PZ. Figure 4 is an example of a spectral map of the entire prostate gland of a man with biopsy-proven PZ and TZ PCa lesions.

**Fig. 4:** T2WI images with spectroscopy grid (middle panel) of a 72-year-old patient with an elevated serum PSA level of 14.5 ng/ml, who was diagnosed with biopsy proven cancer lesions with Gleason 4 + 3 in the left peripheral zone and a Gleason 3 + 3 lesion in the left transition zone. The red circle identifies a voxel in cancer region (right hand side spectrum) and green circle identifies a voxel in normal tissue of the peripheral zone (left hand side spectrum)

The mean and standard deviation values of mp-MRI parameters in TZ cancer and normal tissue are given in Table 3. ADC values derived from DWI measurements were significantly lower in cancerous tissues than in normal tissues (*p* < 0.01). The pharmacokinetic parameters K^trans^, K_ep_ and iAUGC, derived from DCE MRI, increased in cancer tissues compared to normal tissues (*p* < 0.05). The mean values of (Cho + Spm + Cr)/Cit, Cho/Cit and Cho/Cr from the MRSI examinations in cancer ROIs were significantly higher than in normal tissues (*p* < 0.01). There was also a significant difference in all metabolite ratios of cancer compared to normal tissues in PZ (*p* < 0.01).

**Table 3:** Mean ± standard deviation of multiparametric magnetic resonance imaging (mp-MRI) parameters for discrimination of cancer and normal tissue in the central gland

Parameters	Normal	Cancer (low-risk, intermediate-risk and high-risk)	*p-value*
ADC (10^–6^ mm^2^/s)	1112.42 ± 138.83	871.10 ± 149.61	< 0.01
K^trans^ (min^−1^)	0.14 ± 0.08	0.24 ± 0.10	< 0.01
K_ep_ (min^−1^)	0.65 ± 0.38	1.12 ± 0.53	< 0.01
iAUGC (mmol.min/L)	2.61 ± 1.04	3.15 ± 1.31	< 0.05
(Cho + Spm + Cr)/Cit	0.23 ± 0.09	1.60 ± 1.12	< 0.01
Cho/Cit	0.16 ± 0.08	0.82 ± 0.38	< 0.01
Cho/Cr	1.28 ± 0.68	2.94 ± 0.87	< 0.01

*ADC* apparent diffusion coefficient, *K*^*trans*^ the volume transfer constant, *K*_*ep*_ the rate constant , *iAUGC* the area under gadolinium curve, *Cho* choline, *Spm* spermine, *Cr* creatine, *Cit* citrate

### Individual and combined MR imaging metrics to detect cancer tissue

Figure 5 shows ROC curves of final RBF-SVM models for each pair of groups with and without MRSI (left side). These results demonstrated that MRSI significantly improved the AUC (*p* < 0.01) and also sensitivity and specificity (*p* < 0.01) in the detection of TZ cancers (bar charts on right side of Fig. 5). There was no significant difference between AUC, sensitivity and specificity of T2WI + DWI and T2WI + DWI + DCE (*p* > 0.05) and also between T2WI + DWI + MRSI and T2WI + DWI + DCE + MRSI models (*p* > 0.05).

**Fig. 5:** Results of support vector machine analysis to discriminate cancer from normal tissue in the prostate transition zone. Left: ROC plot of combinations of multiparametric MRI values. T2WI + DWI is in blue and T2WI + DWI + DCE in green. Without MRSI is represented by a dashed-line and with MRSI by a solid-line. Only multiparametric MRI parameters with statistically significant differences between cancer and normal tissues (*p* < 0.05) were used for classification. Right: Bar charts of AUC values, sensitivity and specificity of the corresponding RBF-SVM models. McNemar test was used for pairwise comparison of sensitivity and specificities of models and Delong test was calculated for pairwise comparison of AUC of models. **p < 0.01

For models without MRSI, T2WI + DWI achieved the highest AUC, accuracy and specificity at 0.86, 0.83 and 0.85, respectively and the T2WI + DWI + DCE model yielded the highest sensitivity at 0.84. The accuracy and specificity of the T2WI + DWI model was higher than that of the T2WI + DWI + DCE model.

For models including MRSI metabolite ratios that performed significantly better than without these ratios (*p* < 0.05), the T2WI + DWI + MRSI model achieved the highest AUC, accuracy, sensitivity and specificity at 0.99, 0.96, 0.95 and 0.97, respectively. There was no improvement in detection accuracy by adding DCE to the T2WI + DWI + MRSI model. The AUC, accuracy, sensitivity and specificity of all RBF-SVM models are summarized in Table 4.

**Table 4:** Area under receiver operating characteristic curve (AUC) and diagnostic accuracy, sensitivity and specificity of detecting central cancers by T2WI (standardized T2WI signal intensity), DWI (ADC), DCE (K^trans^, K_ep_ and iAUGC) and MRSI ((Cho + Spm + Cr)/Cit, Cho/Cit and Cho/Cr)

Model	AUC (%95 CI)	Accuracy	Sensitivity	Specificity
T2WI + DWI	0.86 (0.75–1.00)	0.83 (111/134)	0.80 (49/61)	0.85 (62/73)
T2WI + DWI + DCE	0.83 (0.70–1.00)	0.80 (107/134)	0.84 (51/61)	0.77 (56/73)
T2WI + DWI + MRSI	0.99 (0.97–1.00)	0.96 (129/134)	0.95 (58/61)	0.97 (71/73)
T2WI + DWI + DCE + MRSI	0.98 (0.95–1.00)	0.95 (127/134)	0.95 (58/61)	0.94 (69/73)

*T2WI* T2-weighted imaging, *DWI* diffusion weighted imaging, *DCE* dynamic contrast enhancement, *MRSI* magnetic resonance spectroscopic imaging, *CI* confidence intervals

### Correlation of MR parameter values with tumor aggressiveness

Correlation coefficients for the normalized T2WI, and the pharmacokinetic DCE parameters K_ep_, and iAUGC with GS risk groups were very low and non-significant (|r|< 0.25, *p* > 0.05). A low, but significant, correlation was found for K^trans^ (r = 0.29, *p* < 0.05). Compared to the DCE parameters, the average ADC demonstrated a better correlation with the different aggressiveness groups (r = -0.51, *p* < 0.01). The (Cho + Spm + Cr)/Cit derived from MRSI had the highest correlation with tumor aggressiveness (r = 0.64, *p* < 0.01). The correlation coefficients of Cho/Cit and Cho/Cr with different risk groups were r = 0.32 (*p* < 0.05) and r = 0.28 (*p* < 0.05), respectively. Figure 6 shows a boxplot representing the ADC and (Cho + Spm + Cr)/Cit parameters for normal, low-risk, intermediate-risk, and high-risk tissues. Higher grade TZ cancer tissue was associated with lower ADC values (Fig. 6A) and higher (Cho + Spm + Cr)/Cit ratios (Fig. 6B).

**Fig. 6:** Box plots of **A** ADC values and **B** (choline + spermine + creatine)/citrate ((Cho + Spm + Cr)/Cit) values of low-risk, intermediate-risk and high-risk transition zone prostate cancer tissues. The correlations with low-risk, intermediate-risk and high-risk prostate cancer tissues were evaluated with Spearman correlation coefficients. MR parameters of ROIs with normal transition zone tissue are shown for comparison (shaded)

K^trans^ and ADC values were used to build RBF-SVM models between different risk groups (normal vs cancer, low-risk vs high-risk cancer, low-risk vs intermediate-risk cancer and intermediate-risk vs high-risk, (*p* < 0.05)). Then, these models were extended by adding MRSI metabolite ratios to the K^trans^ and ADC values. The ROC curve of the final RBF-SVM model for each set of two risk groups was plotted and AUC’s were determined to compare the diagnostic performance of each model (Fig. 7). The results demonstrate that metabolite ratios improve the AUC, sensitivity, specificity and accuracy for the discrimination of low-risk vs high-risk cancer and low-risk vs intermediate-risk cancer groups (right side of Fig. 7). For instance, the AUC in discriminating low-risk from high-risk cancer significantly increased by adding metabolite ratios from MRSI to the combination of ADC and K^trans^ from 0.64 to 0.86 (*p* < 0.01). There was no significant difference between the performance of models for intermediate-risk vs high-risk cancer with and without MRSI metabolite ratios (*p* > 0.05).

**Fig. 7:** Results of support vector machine analysis to separate tumor aggressiveness classes. Left side: ROC curves of the six RBF-SVM models for low-risk vs high-risk cancer, low-risk vs intermediate-risk cancer and intermediate-risk vs high-risk cancer. A leave-one-out cross-validation technique was used for the combined ADC and K^trans^ (dashed line) and all the combined ADC, K^trans^ and metabolite ratios (solid line) with a significant difference between the two groups (*p* < 0.05). Right side: bar charts of AUC values, sensitivity and specificity of the corresponding RBF-SVM models. McNemar test was used for pairwise comparison of sensitivity and specificities of models and Delong test was calculated for pairwise comparison of AUC of models. **p < 0.01 and * *p* < 0.05

## Discussion

A combination of T2WI, DWI and DCE is the most commonly used mp-MRI set in routine clinical exams for the management of patients with localized PCa as defined by PI-RADS V2 guidelines [16]. Numerous studies evaluated a quantitative combination of these mp-MRI methods to investigate their ability for the detection, localization, grading and staging of cancer in the prostate [16–18]. Most of these studies reported poor-to-moderate accuracy and reproducibility of mp-MRI for localization of PCa in TZ as compared to PZ [7, 19–21]. TZ of patients suspected of having PCa frequently contain regions of glandular BPH and stromal BPH, next to other tissues such as (hypertrophic) anterior fibromuscular stroma [22]. In the diagnosis of TZ cancer, T2WI is usually emphasized more than DWI [23]. Because BPH can appear as hyperintense nodules and stromal BPH as hypointense nodules on T2WI, it remains challenging to differentiate TZ cancer from normal tissue using T2WI alone [24]. Combining T2WI and DWI generally improves TZ tumor detection and localization, although these results are variable [21, 25, 26].

Our results indicate that the combination of T2WI and ADC’s derived from DWI exams including high b-value (1600 s/mm^2^), using RBF-SVM classification, improves the diagnostic accuracy of TZ cancer compared to T2WI alone. This result is similar to that reported previously for TZ [19, 27–29]. Some studies demonstrated better results for TZ cancer detection by combining T2WI and higher b-value DWI (b-value = 2000s/mm^2^) [21, 30].

For the combination of T2WI and DCE, some reports suggested a potential value for DCE parameters in the diagnosis of TZ cancer, but other studies failed to find any added benefit [20, 31]. Our results showed no improvement in AUC, accuracy, and sensitivity in detecting TZ cancer by adding DCE to T2WI + DWI. This agrees with studies in which the detection of TZ cancer was not improved by adding DCE to T2WI [31, 32]. However, a quantitative assessment with linear regression indicated that washout in DCE may contribute to detection efficiency [17]. T2WI + DWI + DCE achieved higher sensitivity and lower accuracy and specificity than T2WI + DWI and T2WI + DCE models. This can be attributed to the marked hyper-vascularity of BPH nodules, which can show rapid enhancement as well as early washout. However, together these MRI methods are still limited for accurate detection and localization of PCa in TZ. An alternative approach to this is adding MRSI to mp-MRI exams, as prescribed in the original PI-RADS (V1) guidelines. Our results (Table 4 and Fig. 5) suggest that DCE can be replaced by MRSI using a GOIA-sLASER sequence to detect TZ PCa.

It is well established that MRSI can provide valuable metabolic information for the non-invasive assessment of PCa [10, 11]. Several studies have concluded that adding MRSI to mp-MRI exams improves the diagnostic performance of detecting cancer in TZ [33, 34]. Also in a multi-centre trial MRSI was shown to be able to discriminate between cancer and normal TZ tissues [35]. Most of the previous prostate MRSI studies employed PRESS with standard RF pulses at TE > 100 ms, representing a T2 penalty on all signals of interest. Due to the suboptimal slice selection of standard RF pulses, causing unpredictable lipid signal contamination, and this T2 penalty, the added value of MRSI in mp-MRI of TZ was limited, in particularly when performed without using an endorectal coil [32].

The results of this study demonstrate that metabolic information derived from MRSI using GOIA-sLASER can accurately differentiate among low-risk and clinically significant PCa in TZ. These results also indicate that adding MRSI data, acquired with a GOIA-sLASER sequence, to the routine clinical MRI exam can significantly improve accuracy. The useful role of quantitative MRSI parameters in combination with functional parameters in TZ tumor detection has been acknowledged in the literature [33, 36] Using an RBF-SVM model generated from T2WI, ADC and the metabolite ratios, we obtained high values for AUC, accuracy, sensitivity and specificity for diagnostic separation of cancer from normal. A similar performance was reported for a quantitative study in which TZ PCa was discriminated from normal tissue using an endorectal coil at a TE = 85 ms and combining the Cho/Cr ratio from MRSI and ADC values [17].

In addition to the above, the correlation of mp-MRI parameters with low-risk (GS = 3 + 3), intermediate-risk (GS = 3 + 4) and high-risk (GS ≥ 4 + 3) cancers was investigated. Quantitative T2WI and pharmacokinetic DCE parameters did not correlate with the GS risk groups except for a low correlation with K^trans^. This could be due to heterogeneity in tumor and normal tissue perfusion within TZ. The individual parameters (Cho + Spm + Cr)/Cit and ADC showed a moderate correlation with tumor aggressiveness. However, by combining K^trans^, ADC and metabolite ratios in an RBF-SVM model we found an AUC of 0.86 for the discrimination of low-risk from high-risk cancers.

The identification of low-risk vs high-risk cancers is of clinical importance as it may be used to avoid overtreatment of patients with PCa. Comparable performances in the separation of low from high-risk cancer were obtained in studies of TZ using an endorectal coil and regression models involving ADC or DCE washout and metabolites from MRSI data [17, 37].

It is worth noting that 3D PRESS MRSI has been demonstrated to give reproducible results at 1.5 T with an endorectal coil in a test-retest setting [38]. In later publications it was demonstrated that 3D GOIA-sLASER MRSI is superior to 3D PRESS MRSI [12] and that the former can be applied to the prostate without using an endorectal coil producing reliable metabolic values [39]. One of the limitations of the current study is the relatively small number of intermediate and high grade TZ cancer patients for classification and prediction. Another limitation of this study is that the histopathological classification of lesions is based on a biopsy instead of on whole mount sections.

## Conclusion

This study demonstrated that MRSI with a GOIA-sLASER sequence in combination with structural T2WI and DWI offers a non-invasive and reliable tool to assess cancer tissue in the central prostate gland. We found that DCE has limited value in TZ cancer detection and localization. Although the correlation between cancer aggressiveness and metabolic ratios or ADC values was moderate, the combination of these two enabled a good separation between low-risk and high-risk cancers in TZ.

## Data Availability

The datasets generated during and/or analysed during the current study are available from the corresponding author on reasonable request.

## Abbreviations

3D: Three dimensional
ADC: Apparent diffusion coefficient
AUC: Area under curve
BPH: Benign prostatic hyperplasia
Cho: Choline
Cit: Citrate
Cr: Creatine
CRLB: Cramer–Rao lower bound
CSDE: Chemical shift displacement error
DCE: Dynamic contrast enhancement
DRE: Digital rectal exam
DWI: Diffusion-weighted imaging
FWHM: Full width at half maximum
GOIA: Gradient-modulated offset-independent adiabatic
GS: Gleason score
iAUGC: Area under gadolinium curve
K^trans^: Volume transfer constant
K_ep_: Rate constant
Mp-MRI: Multiparametric MR imaging
MRSI: Magnetic resonance spectroscopic imaging
PCa: Prostate cancer
PSA: Prostate specific antigen
PI-RADS: Prostate imaging reporting and data system
PRESS: Point-resolved spectroscopy
PZ: Peripheral zone
RBF: Radial basis function
ROC: Receiver operator characteristic
ROI: Region of interest
sLASER: Semi-localized adiabatic selective refocusing pulse sequence
Spm: Spermine
SVM: Support vector machine
TRUS: Transrectal ultrasound
TZ: Transition zone
T2WI: T2-weighted imaging
VOI: Volume of interest
